# Problems and Countermeasures of Financial Risk in Project Management Based on Convolutional Neural Network

**DOI:** 10.1155/2022/1978415

**Published:** 2022-03-18

**Authors:** Ran Wei, Dewen Ding

**Affiliations:** ^1^School of Accounting, Shandong Women's University, Jinan, Shandong 250300, China; ^2^School of Computer Science and Technology, Shandong Normal University, Jinan 250358, China; ^3^Shandong Provincial Education Department, Jinan, Shandong 250000, China

## Abstract

Under the background of market economy, engineering projects are faced with a lot of financial risks. If we cannot prevent them effectively, it will undoubtedly bring serious negative impact to the entire engineering management work. Therefore, it is particularly important to actively manage risks, identify and evaluate risks in a timely and correct manner, manage risks efficiently, and minimize risk losses. At the same time, the development of wireless communication technology has brought many new branches of engineering project management. Some problems in the process of risk management are often not handled by traditional empirical calculation or mathematical methods, so it is necessary to find an appropriate way to define and describe the nonlinear relationship between a large number of uncertain causes and risk losses. In order to match the changes in the background of the development of wireless communication technology, this paper studies the financial risk problems and countermeasures in the engineering management of convolutional neural networks. The financial risk prediction model in network engineering management is constructed, and the volume neural network algorithm referenced by it is tested. The test results are highly consistent with the expert assessment. In the research process, the combination of questionnaire survey and mathematical analysis method was adopted, the extreme value of risk factors was determined by questionnaire survey, and then the accuracy of prediction was verified by a mathematical model. After many calculations, it has been proved that the convolutional neural network simulation system based on the scientific node selection method has greatly improved the accuracy of risk assessment.

## 1. Introduction

There are a few studies on engineering risk in my country. From a risk management perspective, most of the research does not discuss it in a detailed and targeted manner but simply generalizes and explains it, some of which may be trivial and overkill without a more detailed investigation [1, 2]. In practice, some technical builders do not understand risk management and do not preidentify and assess project risks [3, 4]. The empirical approach of managers and constructors is effective in risk management, but it is also blind. Some executives do not fully understand the importance of risk management [5, 6]. In addition, it is not enough to supervise the development of the industry in my country alone. Many public work projects have various reasons such as uncertainty of responsibility and authority in the entity management [7, 8]. In recent years, various engineering disasters have been reported by the media, and most of the causes are directly related to poor risk management. This phenomenon should cause us to attach great importance to risk management. Many factors are in a scattered and hidden state at ordinary times, and only when they are triggered and amplified, will they be paid attention to by the construction party. To solve this problem, project management introduces neural network models into the field of risk management. This model imitates the natural neural network of the human body, which can integrate various information in the field on a large scale, and monitor and predict the change of information [9, 10].

In view of the research on engineering risk management, some researchers believe that as engineering work becomes more and more complex, various risks may be faced in the construction process. Strengthening management can effectively predict and avoid possible occurrences in the process of project implementation. They believe that it is very important to choose a scientific decision-making method in risk assessment [11]. My country's research on engineering risk is not very mature, so there are major defects in the selection and application of methods: first, some risk factors or some important factors may be ignored because the selection of risk factors is not sufficient. Quantitative methods also have many subjective factors. The evaluation method established in the evaluation stage is not very scientific. All risk factors are treated equally, and the priorities are indistinguishable. This destroys the foundation of subsequent risk management links and increases the workload of risk management [12]. In terms of financial risk research, some scholars have studied and analyzed the financial risks of my country's pharmaceutical industry enterprises and selected 20 economic indicators in 6 categories such as profit rate, debt service rate, and debt rate risk. Factor analysis was first used to reduce the dimensionality of these indicators, and then a model was created to discover indicators related to a company's financial risk [13]. To sum up, there are many research results on risk prediction, but the application of deep learning in risk prediction needs to be further explored.

This paper studies the financial risk problems and countermeasures in the engineering management of convolutional neural networks. Based on the literature, the financial risk management and financial risk prediction problems in engineering management are analyzed, and then the engineering management based on convolutional neural networks is analyzed. A financial risk prediction model is constructed, then tested, and relevant conclusions are drawn from the test results.

## 2. Research on Financial Risk Issues and Countermeasures in Project Management

### 2.1. Financial Risk Management

#### 2.1.1. Risk Management Usually Including Risk Identification, Risk Assessment, and Risk Management

*(1) Risk Identification.* Risk identification is the premise and prerequisite of risk management. It emphasizes tracking all aspects of construction information and related market changes at any time, and classifying possible risk factors so as to provide methods for risk avoidance or loss reduction in the first time [14]. Risk identification is to analyze the causes of risks by collecting relevant information, and summarizing and classifying data. Identifying all hazards is not easy, and hard-to-identify risks often cause accidental damage.

*(2) Risk Assessment.* Risk assessment is the measurement of risk. That is, through the corresponding assessment of the probability of risk and the size of the loss, the degree of threat to development, the possible damage, and the resulting consequences are analyzed [15]. Factors such as time and location of risk are all related to the level of risk exposure and loss. In order to improve the efficiency of risk management more effectively, it is necessary to pay enough attention to the evaluation work. In this way, when faced with the problem of “choose one of two,” it will not make the wrong decision [16]. If the risk assessment is not accurate enough, the risk management costs will be high and the expected benefits will not be achieved [17]. At this stage, there are more and more models and systems for the scientific development of risk assessment.

*(3) Risk Management.* Risk management is the final stage of risk management. A variety of risk-related factors need to be considered during the practical operation phase: the magnitude, nature, and purpose of the risk. To minimize risks, managers need to choose effective measures to deal with them.

  2.1.2. Characteristics of Risk Management

1. Comprehensive. The risks faced by construction projects are not single but a complex set of intertwined factors. It is necessary to clarify the relationship between various risk factors, effectively understand the factors that lead to risk, and enable staff to develop risk awareness and apply risk concepts in the process of achieving goals.
2. The goal is clear. Risk management has a clear goal, which is to reduce the damage caused by risks to construction projects as much as possible through the identification, assessment, and control of risks.
3. Predictability. The importance of risk management lies in the systematic identification and classification of various risks that have not yet occurred so as to formulate appropriate risk response strategies before they occur to reduce potential losses. The principle is to use systematic analysis to achieve predictive evaluation results.
4. It works. Risk management can maximize low cost management. Calculating additional costs that may arise through risk analysis can help make project budgets more cost effective and avoid concerns about cost overruns.
5. Reliability. Scientific risk management methods are the brainchild of many researchers. They have proposed highly targeted management models for different types of construction projects. This makes the current stage of risk management enter a fairly mature stage, with high reliability.

### 2.2. Financial Risk Prediction in Project Management

#### 2.2.1. Model Prerequisites

Both univariate features and multivariate discrete analysis have high application value. The prerequisite for choosing which model to manage is to see whether it matches the specific conditions of the project. Hypothesis is the most stringent conditional probability model [18, 19]. The two sample sets must have equal covariances, but the explanatory variables need not be normally distributed, and the assumptions are relatively loose [20]. The survival analysis model has loose conditions and needs to bind samples, and there is no requirement for the type of survival function distribution. Artificial neural network models do not require any assumptions.

#### 2.2.2. Model Range

Within the framework of specific construction projects, there are also many model branches. Because of the looser model conditions, survival analysis models are suitable for most data situations. The practical effect of the survival analysis model is very ideal, which can improve the stability of the model [21, 22]. The introduction of the artificial neural network model has brought traditional financial management to a higher level and made up for some of the latter's shortcomings.

#### 2.2.3. Overall Analysis of the Model

In conclusion, the variables selected for discriminant analysis should obey a normal distribution, which is classified according to how many variables are involved. Among them, single variable selects a single economic variable for financial risk prediction, which is simple to operate and has a small workload [23, 24]. Multivariate identification involves the analysis of multiple financial indicators, which requires higher workload and operational complexity, but is more objective, which helps to improve the prediction accuracy of the model.

### 2.3. Convolutional Neural Networks

The function *f*(*x*) represents the nonlinear activation function. The most commonly used functions at this stage are the sigmoid function and the tanh function [25]. The calculation formulas of the two are as follows:

(1) $$\begin{array}{c} F\text{sig}\left(x\right)=\frac{1}{1+1/\gamma^{x}}, \end{array}$$

(2) $$\begin{array}{c} F\;\tan\left(x\right)=\frac{\gamma^{x}-1/\gamma^{x}}{\gamma^{x}+1/\gamma^{x}}, \end{array}$$

where *e* is the logarithm.

From the equation, the method of computing the eigenvalues on the convergence plane can be divided into three steps [26]. First, different convergence kernels converge to the corresponding features of the previous layer; second, the cumulative effect undergoes nonlinearity; third, the activation function acquires the properties of the aggregation layer [27].

### 2.4. Applications of Convolutional Neural Networks

#### 2.4.1. Sparse Connection Method

The sparse connection method changes the traditional hierarchical connection system and adopts the form of local transmission, which greatly improves the speed and accuracy, and also reduces the reflection time of the upper level, making the whole system more efficient. This architecture is inspired by visual effects in biological natural mechanisms; that is, the biological visual analysis of natural images does not process all the information captured by the eye at a specific time but focuses on local regions of the image. Compared with other areas, the elements in this area are more closely related to the subject, so it is easier to attract the subject's attention. At this stage, big data analysis and push are also taking a similar idea.

Therefore, the sparse connection structured in this way will have higher efficiency in the screening and judgment of effective information, thereby simplifying the operation structure of the model and reducing the existence space of errors. After many experiments and comparisons, it is found that the number of parameters collected by the traditional neural network structure is 5 × 3, and the number of parameters collected by the sparse connection architecture is 3 × 3. Under the background that the evaluation results of the two are generally consistent, the sparse connection architecture obviously has a greater advantage.

#### 2.4.2. Weight Sharing

Weight sharing is another important feature of convergent neural networks, which can be clearly explained as follows: the parameters collected from a local area are applied to other secondary areas; that is, the basic unit of the main part will appear multiple times in other areas. If the underlying features of the image are repeated, edges, angles, lines, etc. are more likely to be repeated in different positions. So, if you apply the same filter to the whole property graph, you will get all the properties that satisfy the specific properties of the property graph. The Sobel kernel commonly used at this stage is developed following this assumption. From another perspective, convergent neural networks have a certain tolerance for linear transformations because weight sharing can detect the same patterns at different locations in the data.

## 3. Financial Risk Prediction Model in Engineering Management Based on Convolutional Neural Network

### 3.1. Principles of Selection of Risk Indicators

1. Systematic principles. The scope and relevance of index selection need to be carefully considered when constructing risk metrics.
2. The content of construction projects is very complex, and any content may breed risks with changes in the objective situation. If the key points are ignored and the overall consideration is taken, it will not only reduce the vigilance of enterprises for serious risks but also involve too much energy. Therefore, when building a financial risk prediction model, we must carefully select those key nodes in the financial operation process and adopt a hierarchical and focused detection mode. This allows managers to monitor potential financial risks to project operations [28].
3. Principle of validity. The core of risk management is ex ante management. A successful early warning effectively anticipates all aspects of the project process, not just on-site inspections or postmortems. Therefore, the construction management party should forecast the development prospects of the project according to the actual situation of the project, combined with national policies and market demand. A scientific index system is built, and the risk of the project is prewarned by assigning the interval value of each index.
4. Functional principle. Establishing an early warning model of financial risk is the basis for project risk management. Therefore, when designing the early warning indicator system, the feasibility of the actual operation of the indicators should be considered, including the early warning of relevant financial indicators and a simple understanding of the indicators. Metrics that are difficult to obtain or remain controversial in the theoretical realm should be handled with caution.

### 3.2. Selection of Risk Indicators

Risk factors represent the risks of a project. In the stage of determining the financial risk management model, the risks of the entire project are divided into three categories: “project engineering,” “project environment,” “project constraints,” and corresponding 13 elements. Each element is divided into features, each of which represents a risk factor. Under normal circumstances, there are more than 50 categories of risk factors that can be promoted by construction projects, but due to different projects, the risks of each category have different impacts on the project. As we take, for example, the “security” risk factor, a project involving online transactions where security is a top priority. However, typical projects do not require high levels of security. Multiple studies have confirmed that even supposedly secondary factors can sometimes become significant risk factors, resulting in measurements often strongly interfered with by nonessential factors. This requires us to strictly verify the validity of the risk factors when designing the model. The first step is to verify the validity of the risk factors introduced by the model. Here, this paper conducted in-depth interviews with 10 experts, including project managers, enterprise project managers, and customer project managers, through a questionnaire survey. In the questionnaire, there is a total of 54 questions corresponding to the common risk types at this stage.

Again, the questionnaire contains quantitative questions. Respondents simply answered “yes” or “no.” The occurrence of this risk factor is quantified based on the specific state of the response. The contribution of the question is positive if the answer to the question helps to increase the likelihood of the risk factor, and negative otherwise. The exact number depends on the problem with each element. If the risk factor has four first-level questions, the contribution of each question is +0.25 or −0.25. For some Level 1 questions with Level 2 questions, the specific contribution is also calculated based on the number of Level 2 questions.

Given the varying importance of each risk factor, it is not possible at this stage to rely solely on the quantification methods described above. For simplicity, this paper stipulates that if the product of factor quantification and factor significance quantification exceeds 0.3, the factor is identified as a high-risk factor and needs attention.

### 3.3. Implementation of Convolutional Neural Networks

Since this article only looks at the impact of historical data on the value at a specific point in time, the dimension of the data is one dimensional. Such a design optimizes the architecture of the skilled neural network and effectively improves the working efficiency of the convergence kernel. The optimization of the architecture is the significant difference between this design and the traditional convergent neural network structure. Experiments show that the difference in the number of convergence layers and sampling layers will have a great impact on the size of the convolution kernel, which in turn will interfere with the experimental results. Therefore, this study assumes a fixed proportion of the volume of each convolution kernel during the convolution process. The convergence kernel number of the second convergence stage is twice the number of the convergence kernel number of the first convergence stage, and the downsampling is the same. The convergent neural network prediction model consists of an input layer, two convergent layers, and a five-level network consisting of a downsampling plane and a single-layer perceptron.

## 4. Test of Convolutional Neural Network

### 4.1. The Displacement Factor *n* of the Activation Function

According to the constantly changing value of the algorithm shift factor *n*, the influence of these expressions on the convergence speed of the algorithm is studied. The results are shown in Table 1.

It can be seen from Table 1 that if *n* = 0, it is the initial activation function, and the inertia of repeated values is enhanced. If *n* < 0, the number of iterations is gradually relatively stable, and the reset value decreases slowly. In sharp contrast, in the interval of *n* > 0, as the value of *n* increases, the number of iterations increases sharply, and the reduction curve of the repetition value is very obvious. This shows that if a scientific displacement factor is selected in the experiment, the convergence speed of the algorithm can be effectively improved, and the working time can be greatly reduced.

### 4.2. Optimizing the Number of Convolutional Layer Nodes

Although from a theoretical point of view, the three-level neural network is sufficient to support the existing risk prediction model, in practice, this three-level system has certain shortcomings. The most typical case is that when faced with a large number of convolutional layer nodes, the calculation results often deviate. Therefore, the determination of the number of nodes is very important for model operation. It is necessary to find the balance between the computing power and generalization ability of the neural network according to the specific needs of the model. To achieve this goal, the study chooses the golden ratio method to determine the number of nodes in the cohesion layer. The method has low cost, high efficiency, and strong practicability. The main tasks of the optimization algorithm are as follows:

In this article, the data are sorted correctly. The input layer has 16 nodes, and the output layer has 1 node.

For complete comparison and analysis, all training results in the convolutional layer nodes [11, 16] are shown in Table 2.

It can be seen from Table 2 that when the number of nodes is 18, the total error of the network is the smallest and the approximation accuracy is the best.

Training results from Table 3 show the simulation results of the five sets of stests without training. This is consistent with the expert evaluation results shown in Table 3, and the comparison of the results is shown in Figures 1 and 2.

As can be seen from Figure 1, there is little difference between the training result and the expected result. Among the 10 comparison groups, 60% of the groups have more of the former, indicating that the prediction of the training result is more rigorous and the sensitivity to risk factors is higher.

It can be seen from Figure 1 that after calculation, the simulation results and the expert results have a high degree of similarity, and the deviation of the results is within 1%, which proves that it has a very high accuracy.

It can be seen from Figure 2 that determining the number of nodes through the golden ratio method has a very positive effect on improving the accuracy of the risk early warning mechanism. The test set simulation results are based on expert estimates, and the accuracy percentage is as high as 99.3%, so the number of convolutional layer nodes can be optimized using the golden ratio method.

## 5. Conclusions

The financial risk of construction projects is an issue that construction units must pay attention to. This paper studies the financial risk problems and countermeasures in the engineering management of convolutional neural networks. After using the questionnaire survey method to determine the risk indicators, a simulation analysis model is constructed, which is based on the sparse connection method and is more efficient and accurate than the traditional connection method. In future research, we will continue to optimize the model along this line of thought to reduce possible errors as much as possible.

## Figures and Tables

**Figure 1:** The number of hidden layer nodes is 16, and the number of training times is *N* = 12000.

**Figure 2:** Simulation results of five sets of tests without training.

**Table 1:** The influence of expression on the speed of algorithm convergence.

*n* value	−2	−1	0	1	2	3	4	5
Error	0.003	0.003	0.005	0.005	0.005	0.007	0.007	0.007
Number of iterations	1669	1618	1499	1318	1129	921	633	392

**Table 2:** All training results in the convolutional layer nodes [11, 16].

Number of nodes	Number of iterations	Total error *E*	Number of nodes	Number of iterations	Total error *E*
11	998	0.0059	19	1000	0.0016
12	871	0.008	20	992	0.0049
13	996	0.012	21	988	0.0231
14	729	0.00094	22	983	0.0072
15	997	0.0061	23	756	0.0091
16	281	0.0078	24	976	0.0458
17	995	0.0009	25	975	0.0072
18	997	0.00058	26	991	0.0095

**Table 3:** Simulation results of five sets of tests without training.

Item number	11	12	13	14	15
Training result	0.669	0.438	0.487	0.359	0.687
Expected output	0.677	0.415	0.485	0.368	0.679
Simulation results	Fair risk	High risk	High risk	High risk	Fair risk
Expert results	Fair risk	High risk	High risk	High risk	Fair risk

## Data Availability

The datasets used and/or analyzed during the current study are available from the corresponding author on reasonable request.
